# Sports Auxiliary Training Based on Computer Digital 3D Video Image Processing

This article has been retracted.

**DOI:** 10.1155/2022/2105790

**Published:** 2022-01-10

**Authors:** Saisai Xu

**Affiliations:** Henan University of Economics and Law, Zhengzhou 450016, China

## Abstract

With the continuous development of social economy, sports have received more and more attention. How to improve the quality of sports has become the focus of research. The computer digital 3D video image processing is introduced in this paper, taking shooting as the starting point, in which computer digitization technology is used to collect images of sequence targets through combining the operation flow of shooting, monitor the results and data of shooting and process 3D video images, conduct the analyze and mine according to the corresponding statistical processing results, and evaluate the corresponding training. The simulation experiment proves that the computerized digital 3D video image processing is effective and can scientifically support sports-assisted training.

## 1. Introduction

With the development of social economy, sports have received more and more attention as an important way for people to exercise. In competitive competitions, how to improve the quality and effectiveness of sports players is extremely important [1, 2]. Traditional training methods are usually dominated by coaches, and they are judged and corrected through experience to achieve the integration of training rhythms and methods [3, 4]. But, most sports have strong requirements for athletes' balance, attention, coordination, and sense of time. Therefore, how to quantitatively improve athletes' training performance is the focus of further investigation [5, 6]. The development of computer technology has led to the development of many assistive technologies, and the computer-related technologies have been introduced into sports training within the industry to further improve the summary of exercise rules and exercise effectiveness, so as to achieve scientific and effective sports training [7, 8].

During the process of sports training, computer technology can replace a variety of roles and functions, such as simulating sports and capturing corresponding 3D simulation sports (boxing, table tennis, etc.); 3D simulations and emulations of high jump actions are performed through 3D movies to realize training analysis and analyze the authenticity of the athlete's movement [9–11]. Therefore, in the actual sports training process, it is necessary to integrate image capture and three-dimensional simulation. Through image processing, cleaning, and analysis, the three-dimensional sports simulation of athletes is realized. At the same time, the corresponding dynamic data and equations are used to simulate athletes' movements, realize synchronous perspective and synchronous training according to training requirements and needs, and provide reference for sports training [12–14].

For shooting sports, it pays more attention to attentiveness, critical state, etc. Traditional training usually uses visual artificial judgment. In actual training, there are often the problems of inaccurate judgments, long time-consuming, and inability to analyze relevant data. Therefore, in response to this need, the computer digital 3D video image processing is introduced in this paper, computer images are used to identify the shooting target ring through the analysis of the shooting movement process, and the shooting results parameter changes are calculated real time to achieve the evaluation of the training results, aiming at providing an auxiliary reference for sports training, so as to improve the quality and effect of training.

## 2. Computer Digital 3D Video Image Processing

For computer digital 3D video image processing, the specific principle is shown in Figure 1. First, the simulated data need to be visualized. Secondly, according to the needs, the typical characteristic area shall be selected as the relevant sample data for classification. These samples are stored in the corresponding training network to save the results, and corresponding data recognition is performed through feature acquisition [15, 16]. During the actual processing process, feature samples can be selected according to corresponding needs and demands, and training iterations can be performed to realize feature visualization.

### 2.1. Feature Detection and Recognition

For feature detection and recognition, real-time interactive processing is required. The feature detection and recognition algorithm is carried out on the CPU, and in order to improve the speed, the method of taking the area of the critical point as the candidate unit is adopted. In order to realize the real-time interaction of feature detection and recognition, this paper designs a GPU-based feature detection and recognition algorithm. The basic idea is to convert the flow field into texture fragment blocks and use the high parallel characteristics and programmability of GPU to convert BP neural network feature recognition into processing texture fragments. The basic flow is shown in Figure 2. The algorithm mainly includes the following steps:

**Step 1 .**

Texture conversion: it is responsible for converting the flow field data into a color texture that is easy to process by the GPU.

**Step 2 .**

GPU processing: it is responsible for feature recognition of the area where the current fragment is located.

**Step 3 .**

Saving the results: it is responsible for reading the recognition result from the GPU and saving it to the corresponding data structure.

Because the GPU feature recognition process is a parallel process, this paper does not adopt the critical point region candidate unit method, but uses the sequential traversal method. The reason is analyzed as follows: When using the critical point candidate unit method or the traversal method on the GPU, assuming that the texture conversion process time is ${\bar{T}}_{1}$ and *T*_1_, the GPU processing process is ${\bar{T}}_{2}$ and *T*_2_, and the result saving process is ${\bar{T}}_{3}$ and *T*_3_, the entire pipeline The processing time is $\bar{T}={\bar{T}}_{1}+{\bar{T}}_{2}+{\bar{T}}_{3}$ and *T*=*T*_1_+*T*_2_+*T*_3_, respectively. Since Step 1 and Step 3 require the same time for the two methods, namely ${\bar{T}}_{1}=T_{1}$, ${\bar{T}}_{3}=T_{3}$, the length of the pipeline processing time depends on ${\bar{T}}_{2}$ and X*T*_2_. The critical point area candidate unit method needs to discriminate the fragment type in the fragment shader. If the current fragment corresponds to the critical point, then the identification judgment is performed; otherwise, the process is skipped. Let's suppose that the fragment shader *F*_*i*_ corresponds to the critical point fragment type, and the processing time is ${\bar{T}}_{F_{i}}$, and the fragment shader *F*_*j*_ corresponds to the non-critical point type, and the processing time is ${\bar{T}}_{F_{j}}$. Although ${\bar{T}}_{F_{i}}<{\bar{T}}_{F_{j}}$, because the GPU is a parallel processing process, the shader with the longest calculation time among the fragment shaders constitutes the bottleneck of the recognition algorithm, thus ${\bar{T}}_{2}=\max\left({\bar{T}}_{F_{i}},{\bar{T}}_{F_{j}}\right)={\bar{T}}_{F_{j}}$. Similarly, there is *T*_2_=max(*T*_*F*_*i*__), 0 ≤ *i* ≤ *N* for the traversal method, where *T*_*F*_*i*__ is the processing time of each fragment. Because the segment type judgment process sentence is added in the critical point area candidate unit method, there must be ${\bar{T}}_{2}=\max\left({\bar{T}}_{F_{i}}\right)>\max\left(T_{F_{i}}\right)=T_{2}$, so $\bar{T}>T$. That is, in the GPU processing process, the speed of the traversal method is better than that of the critical point candidate unit method. (Algorithm 1).

First, obtain the node data of the characteristic area according to the current texture coordinates, then perform the characteristic recognition calculation, and set the current fragment color according to the recognition result. The implementation code of the feature recognition process is basically the same as that on the CPU, but the texture-speed reverse calculation is first required; in addition, to ensure that the texture conversion process does not lose data accuracy, the texture format uses a 32 bit floating point type.

This paper also uses the pressure field data to correct the characteristics of the BP neural network. In the experiment, the characteristics of cyclones and anticyclones were mainly extracted, and cyclones and anticyclones correspond to the low and high pressure centers in the pressure field, respectively. There is a pressure *P* ≤ *P*_threshhold_ for the center of the cyclone and *P* ≥ *P*_threadhold_′ for the center of the anticyclone. For wind field data, assume that the position obtained after feature detection using BP neural network is *P*_*i*_, and the position obtained after detecting the corresponding pressure field data using the pressure amplitude method is *P*_*i*_′. If *D*(*P*_*i*_, *P*_*i*_′) ≤ *d*_threshhold_, the detection result is considered correct and output *p*_*i*_; otherwise, the detection result is considered to be wrong, where *d*_threshhold_ is the Euler distance error threshold.

### 2.2. Multiresolution Rendering

Due to the unevenness of the image, an octree is needed to divide the corresponding space. The specific principle is shown in Figure 3.

Voronoi diagram is a space division structure generated based on the principle of nearest neighbors, and its definition is as follows: suppose S is a two-dimensional plane *q* which is any geometric point on S, and *XO*={*O*_1_, *O*_2_,…, *O*_*n*_},  *n* ≥ 3 is a set of discrete points on the Euclidean plane. The area *V*(*O*_*i*_) is a set that satisfies the following conditions: *V*(*O*_*i*_)={*p|p* ∈ *S*,  and *d*(*p*, *O*_*i*_) ≤ *d*(*p*, *O*_*j*_), *j* ≠ *i*, *j*=1,2,…, *n*}, then *V*(*O*_*i*_) is called the Voronoi area associated with the object *O*_*i*_, and *O*_*i*_ is called the growth object of this area. Let *V*={*V*(*O*_1_), *V*(*O*_2_),…, *V*(*O*_*n*_)}; call *V* the Voronoi diagram on S generated by O. The Voronoi diagram technology is spatially divided to form a polygon set, where each polygon area corresponds to a point target. The distance from each point of the polygon to the corresponding point target is smaller than other point targets. Voronoi diagram can be divided into vector method and grid method according to its generation method, considering the experimental data as a regular grid structure.

A feature-based Voronoi diagram data organization method is proposed based on the grid method in this paper. The steps are as follows:

**Step 4 .**

According to the chessboard distance in Figure 4, extract the corresponding point distance definition.

**Step 5 .**

Local distance propagation calculation is performed for each point target in turn, as shown in the following formula:

(1) $$\begin{array}{c} D\left(i,j\right)=\min\left[D\left(i-1,j-1\right)+1,D\left(i-1,j\right)+1,\right)\\ D\left(i-1,j+1\right)+1,D\left(i,j-1\right)+1,D\left(i,j\right),D\left(i,j+1\right)+1,\\ D\left(i+1,j-1\right)+1,D\left(i+1,j\right)+1,D\left(i+1,j+1\right)+1. \end{array}$$

The distance from the surrounding nodes to the point target is calculated. In Algorithm 1, *D*(*i*, *j*) represents the distance from the node with the serial number (*i*, *j*) to a certain point of target.

**Step 6 .**

According to Figure 5, organize each feature area and adjacent area nodes into a tree structure, which is called a feature tree. If the superscript is used to indicate the layer number of the node in the feature tree, the subscript indicates the sequence number in the layer, such as *N*_*i*_^*m*^ represents the *i*-th node in the *m*-th layer of the feature tree, then the specific construction process of the feature tree is as follows:

**Step 7 .**

Initialize the root node and set the child nodes to be blank.

**Step 8 .**

Iterate 2.1–2.3 until all image processing is completed.

**Step 9 .**

Create a new node *N*_*i*_^1^. Set the corresponding attributes according to the feature category, and set the node as the *i*-th child node of *R*.

**Step 10 .**

Create a new node posture_1_(*t*_1_)=〈*p*_0_^1^(*t*_1_), *q*_0_^1^(*t*_1_),…, *q*_*n*_^1^(*t*_1_)〉 and join the feature tree as the first child node of the node posture_2_(*t*_2_)=〈*p*_0_^2^(*t*_2_), *q*_0_^2^(*t*_2_),…, *q*_*n*_^2^(*t*_2_)〉; obtain the nodes with a distance of *D* ≤ 1 in the graph as child nodes and join the node *q*_0_^1^(*t*_1_) in turn, as shown in Figure 5.

**Step 11 .**

Obtain the neighboring area nodes in the distance graph 2≤*D*≤3, form groups in turn according to the screening scale factor *a*, and filter out the parent nodes *q*_0_^2^(*t*_2_) to join the nodes dist(*q*_0_^1^(*t*_1_), *q*_0_^1^(*t*_2_))=‖log((*q*_0_^1^(*t*_1_))^−1^ × *q*_0_^2^(*t*_2_))‖ according to the screening rules.

For the node screening rule for neighboring area, the method of taking the minimum dimension node is adopted for the experiment in this paper, that is, if the neighboring area node group *M* contains nodes *q*_*i*_^1^(*t*) and *q*_*i*_^2^(*t*), and *r*_*i*_^1^(*t*), then *r*_*i*_^2^(*t*) is selected [17, 18]. After adopting the feature tree method, any feature area corresponds to a unique feature tree subnode, which effectively solves the problem of low efficiency in drawing the feature area when the data field is represented by an octree. The generation and extinction of time-varying field features only correspond to the addition and deletion of a single node in the feature tree. The data structure is easier to maintain. After the feature tree and the global octree are generated, the fisheye view technology is used for multiresolution rendering. The fisheye view technology was first proposed by Furnas. Its basic idea is to display fine-grained information to the user's attention area and coarse-grained information to the background area. After obtaining the feature tree and the global octree, the multiresolution rendering process mainly includes two steps: (1) drawing the nodes in the global octree according to the background field detail control parameter *β*; (2) drawing the corresponding nodes in the feature tree. In order to ensure the authenticity of the visualization of the data field, the original image data are restored appropriately by keeping the data visualization graphs of the focus area and the background area in the same size.

## 3. Visual Aid Training System

For shooting sports training, it can rely on the computer to interpret and read the shooting indication results and meanwhile realize the shooting process backtracking, accounting shooting distribution law, shooting deviation error, and historical shooting data analysis, through the overall analysis of these data; to achieve the assistance of sports training, the specific system block diagram is shown in Figure 6.

By setting up multiple 3D camera instruments, the target image can be collected, and the multiple processing results and data of the shooting location can be monitored. After the computerized collection of multiple 3D images, the unified processing of video data is realized, and finally 3D image preprocessing is realized, such as deformation correction, image segmentation, image calculation, target recognition, and orientation determination, which are processed according to the corresponding results before the shooting data are obtained.

For the processing of the target image, the recognition, statistics, and analysis of the shooting target can be realized. Meanwhile, the deviation calculation is carried out according to the existing design results, and the corresponding shooting correction is given. Ultimately, the quality and effectiveness of shooting training are improved.

## 4. Shooting Data Processing

For shooting data processing, it mainly analyzes and recognizes the digitalized 3D video image, calculates the corresponding shooting ring number, and realizes the unification and display of the results. 3D video image data processing can be divided into image filtering, geometric correction, image segmentation, calculation processing, data storage, and other steps. The specific processing is shown in Figure 7.

The preprocessing of the image is mainly realized by performing grayscale change and filtering processing on the 3D video image. The purpose of the image grayscale transformation is to reduce the dimension of the image data and improve the processing speed. The role of image filtering is to eliminate noise signals in the image and improve the reliability of subsequent processing. Currently, commonly used image processing algorithms are generally applicable to RGB images. Because the target is simple and the shape is basically fixed in the image processing of this system, the processing is performed on grayscale images.

### 4.1. Image Pretreatment

The 3D video image *I*_0_ (RGB) is transformed into a grayscale image I through preprocessing, specifically as shown in the following formula:

(2) $$\begin{array}{c} I\left(x,y\right)=0.299I_{0}\left(r,x,y\right)+0.587I_{0}\left(g,x,y\right)+0.114I_{0}\left(b,x,y\right), \end{array}$$

where *I* (*x*, *y*) is the gray value of the gray image at the coordinates (*x*, *y*), *I*_0_(*r*, *x*, *y*) is the gray value of the red component of the RGB image at the coordinates (*x*, *y*), and *I*_0_(*g*, *x*, *y*) is the gray value of the RGB image at the coordinates (*x*, *y*). The gray value of the green component at the coordinates (*x*, *y*) and *I*_0_(*b*, *x*, *y*) is the gray value of the blue component of the RGB image at the coordinates (*x*, *y*).

Equation (2) is generally used in grayscale conversion occasions, but for images with different tones and brightness, the 3D images obtained are different. Under certain circumstances, the 3D image features obtained are not necessarily the most prominent. Therefore, for the specific environment generally adopts the weighted summation method to calculate, the specific is shown in the following formula:

(3) $$\begin{array}{c} \left\{\begin{array}{c} I\left(x,y\right)=w_{1}I_{0}\left(t,x,y\right)+w_{2}I_{0}\left(g,x,y\right)+w_{3}I_{0}\left(b,x,y\right)\\ w_{1}+w_{2}+w_{3}=1 \end{array}\right., \end{array}$$

where *w*_1_, *w*_2_, and *w*_3_ are the weights of the RGB components of the in-color image, which can be obtained through experiments.

Suppose the image weighted filtering template is shown in the following formula:

(4) $$\begin{array}{c} \left\{\begin{array}{c} h_{l}=\left[\begin{array}{ccc} w_{11} & \cdots & w_{1l}\\ \vdots & \; & \vdots \\ w_{l1} & \cdots & w_{ll} \end{array}\right]\\ \sum w_{ij}=1 \end{array}.\right. \end{array}$$

The image weighted filtering algorithm is shown in the following formula:

(5) $$\begin{array}{c} I^{\prime }\left(x,y\right)=\sum \sum w\left(x+i,y+i\right)I\left(x+i,y+j\right),\\ i\in \left[-\frac{\left(l-1\right)}{2},\frac{\left(l-1\right)}{2}\right],\;i\in Z,\\ j\in \left[-\frac{\left(l-1\right)}{2},\frac{\left(l-1\right)}{2}\right],\;j\in Z, \end{array}$$

where *w*(*x*+*i*, *y*+*j*) is the element value of *h*_*l*_ at (*x* + *i*, *y* + *j*).

Generally, *w*_*ij*_=*w*_*i*′*j*′_=1/*l*^2^ is taken.

### 4.2. Image Segmentation and Model Correction

On the basis of target determination, the single-threshold segmentation method is used for calculation, and the specifics are shown in the following formula:

(6) $$\begin{array}{c} B\left(x,y\right)=\left\{1,I^{\prime }\left(x,y\right)\geq G_{th}\right\},\\ 0,I^{\prime }\left(x,y\right)<G_{th}, \end{array}$$

where *B* is the segmented binary image, and *G*_*th*_ is the segmentation threshold.

In order to further quantitatively calculate and simulate and realize the effectiveness of recognition and calculation, the model replaces the 3D video image and integrates the actual target, which can not only reduce the workload but also reduce the corresponding interference, to achieve accurate simulation. Therefore, the image needs to be segmented first to realize the effective identification of the position of the ring.

By dividing the target, the center and the ring are distinguished, and the side view of the target is realized, and the distortion of the 3D video image is further corrected to obtain a more accurate target model. The specific imaging diagram is shown in Figure 8.

Due to the deviation between the position of the equipment and the target, there will be deformation when acquiring images. As shown in Figure 8, the larger the included angle *θ*, the greater the deformation may be.

## 5. Computer-Aided Training Simulation Experiment

After obtaining the data of a single shot, the system can perform microanalysis according to the characteristics of the detected data and after a complete shot, according to the data distribution characteristics and changes. Meanwhile, it can also analyze the changes in athlete performance based on the changes in historical data, evaluate the training effects of athletes and coaches, and give reference training programs based on the characteristics of the data.

### 5.1. Single Data-Aided Training

The calculation of the correction variable is to give a reference correction value based on the current deviation and the last deviation. Under normal circumstances, it is considered that this shooting is the result of the correction based on the previous shooting data, and the correction deviation is calculated according to the theoretical correction situation, and then the appropriate correction plan is estimated based on the current deviation. If the current shot is the first shot, the data at the center position is the last shot data, and the deviation caused after correction is not made. After the callback, there is a system deviation, so the last excellent target is the adjustment point for adjustment.

### 5.2. Complete Process Assisted Training

Suppose that 10 shots have been completed, and the ordered dataset is *C*={*c*_1_, *c*_2_,…, *c*_10_}; according to the dataset, the ring count change, the position change, the bullet point distribution, the data validity change, and the bullet point system deviation are macro analyzed, and the bullet point dispersion assessment is performed.

#### 5.2.1. Analysis of Data Changes

Through the bullet point data curve, you can observe the changes in the athlete's performance during the entire shooting process, analyze the best and worst points of the state, and provide a reference for the adjustment of the state during the shooting process.

#### 5.2.2. Analysis of Data Statistical Characteristics

The analysis of the statistical characteristics of the data includes the deviation data of the average center point, the statistical circle coordinates and radius of the bullet point set, the dispersion of the data, and the credibility of each data. The center point deviation data is calculated using the mean value of the number of points.

(7) $$\begin{array}{c} \left\{\begin{array}{c} r_{c}=\frac{1}{10}\sum_{i=1}^{10}r_{i},\\ \theta_{c}=\frac{1}{10}\sum_{i=1}^{10}\theta_{i}. \end{array}\right. \end{array}$$

The credibility of the data can be calculated by using the distance between the shooting point and the statistical circle. The closer to the statistical circle center, the higher the credibility of the shot. The farther away from the statistical circle, the lower the credibility of the shot.

#### 5.2.3. Auxiliary Training

The auxiliary training content mainly includes the following:

- Correction of system deviation
- Psychological adjustment reference during shooting
- Reference for posture adjustment during shooting
- Reference for breathing adjustment during shooting
- Suggestions for further improving performance

### 5.3. Tracking and Evaluation of Training Process

The evaluation of the training process includes two levels: athletes and coaches.

#### 5.3.1. Evaluation of the Athlete's Training Process

If the long-term training does not significantly reduce this deviation and shows regular changes, the training method or the athlete's suitability for the sport should be reassessed.

#### 5.3.2. Evaluation of Coach Training Process

In addition to the abovementioned auxiliary training, the auxiliary training system can also statistically analyze the impact of shooting performance and other factors.

- The correlation between shooting performance and shooting environment temperature
- The correlation between shooting performance and sunny and rainy
- Changes in shooting performance with the four seasons
- The correlation between shooting performance and time period, etc.

The specific analysis of the abovementioned situation provides a reference for enhancing the strengths and avoiding weaknesses and strengthening the training purposefully.

Assuming that there are two action segments mi(t) and m2(t), they can be connected into a new action sequence using motion mirroring and motion transition techniques. The last posture of m1(t) and the first posture of m2(t) are set to be

(8) $$\begin{array}{c} {\text{posture}}_{1}\left(t_{1}\right)=\langle p_{0}^{1}\left(t_{1}\right),q_{0}^{1}\left(t_{1}\right),\ldots ,q_{n}^{1}\left(t_{1}\right)\rangle ,\\ {\text{posture}}_{2}\left(t_{2}\right)=\langle p_{0}^{2}\left(t_{2}\right),q_{0}^{2}\left(t_{2}\right),\ldots ,q_{n}^{2}\left(t_{2}\right)\rangle . \end{array}$$

According to the difference dist(*q*_0_^1^(*t*_1_), *q*_0_^1^(*t*_2_))=‖log((*q*_0_^1^(*t*_1_))^−1^ × *q*_0_^2^(*t*_2_))‖ between the direction |*Z*_2_ − *Z*_1_| and |*Z*_3_ − *Z*_1_| to determine whether the action m2(t) needs to be mirrored, the result may still be recorded as m2(t).

Assume that the long side of the virtual trampoline is consistent with the *X* direction, and the wide side is consistent with the *Z* direction, and its coordinate system OXY B is defined according to the right-handed system, and its initial position is assumed to coincide with the global coordinate system. Select the three vertices *p*_1_(*u*_1_, *v*_1_), *p*_2_(*u*_2_, *v*_2_), and *p*_3_(*u*_3_, *v*_3_) of the trampoline from the training video, and assume that *p*_2_ is the common vertices of the long side and the wide side, then the camera orthogonal projection model is shown in the following formula:

(9) $$\begin{array}{c} \left(\begin{array}{c} u\\ v \end{array}\right)=s\left(\begin{array}{ccc} 1 & 0 & 0\\ 0 & 1 & 0 \end{array}\right)\left(\begin{array}{c} X\\ Y\\ Z \end{array}\right). \end{array}$$

The points *p*_1_, *p*_2_, and *p*_3_ can be mapped to the points *P*_1_ (*X*_1_, *Y*_1_, *Z*_1_), *P*_2_ (*X*_2_, *Y*_2_, *Z*_2_), and *P*_3_ (*X*_3_, *Y*_3_, *Z*_3_) in the three-dimensional space, respectively, and the relative depth |*Z*_2_ − *Z*_1_| and |*Z*_3_ − *Z*_1_| can be solved, so as to determine the location of the virtual shooting. The simulation experiment results show that the computer digitized 3D video image is effective.

## 6. Conclusions

Physical training is an important way and means to improve sports performance. Therefore, reasonable and effective physical training is extremely important. Relying on computer digital 3D video image processing, the assistance of the design training system is achieved through combing the shooting process. Through the analysis of 3D image processing, data processing and analysis under different series of shooting levels are realized to achieve data statistics and mining and finally provide support for sports training. The results of the simulation experiment show that the computer digitized 3D video images are effective and can support sports-assisted training.

## Figures and Tables

**Figure 1:** Principle of multiresolution visualization.

**Figure 2:** GPU feature recognition algorithm flow chart.

**Figure 3:** The feature area is located in the octree partition subspace.

**Figure 4:** Checkerboard distance.

**Figure 5:** Feature tree structure based on Voronoi diagram.

**Figure 6:** Computer vision aided training system.

**Figure 7:** Principles of shooting data processing.

**Figure 8:** Schematic diagram of imaging.

**Algorithm 1:** Algorithm 1 Feature detection and recognition algorithm.

## Data Availability

Data sharing is not applicable to this article as no datasets were generated or analyzed during the current study.

## References

[1] Zhang C., Li M., Wang H., Wang N. (2021). Auxiliary decision support model of sports training based on association rules. *Mobile Information Systems*.

[2] Wu Y., Song Y., Huang H., Ye F., Xie X., Jin H. (2021). Enhancing Graph Neural Networks via auxiliary training for semi-supervised node classification. *Knowledge-Based Systems*.

[3] Zhou M., Long Y., Zhang W. (2021). Adaptive genetic algorithm-aided neural network with channel state information tensor decomposition for indoor localization. *IEEE Transactions on Evolutionary Computation*.

[4] Kurihara K., Imai A., Seiyama N. (2019). SMPTE periodical—automatic generation of audio descriptions for sports programs. *SMPTE Motion Imaging Journal*.

[5] Urban J., Decker J., Peysson Y. (2011). A survey of electron Bernstein wave heating and current drive potential for spherical tokamaks. *Nuclear Fusion*.

[6] Prieto Saborit J. A., del Valle Soto M., González Díez V. (2010). Physiological response of beach lifeguards in a rescue simulation with surf. *Ergonomics*.

[7] Thng S., Pearson S., Keogh J. (2019). Correction to: relationships between dry-land resistance training and swim start performance and effects of such training on the swim start: a systematic review. *Sports Medicine*.

[8] Bergeron M. F. (2015). Training and competing in the heat in youth sports: no sweat?. *British Journal of Sports Medicine*.

[9] Brenner J. S. (2016). Sports specialization and intensive training in young athletes. *Pediatrics*.

[10] Yz A., Ctcb C., Ngma D. (2020). The effects of visual training on sports skill in volleyball players. *Progress in Brain Research*.

[11] Ciolac E. G., Rodrigues-Da-Silva J. M. (2016). Resistance training as a tool for preventing and treating musculoskeletal disorders. *Sports Medicine*.

[12] Baugh C. M., Kroshus E., Lanser B. L., Lindley T. R., Meehan W. P. (2020). Sports medicine staffing across national collegiate athletic association division I, II, and III schools: evidence for the medical model. *Journal of Athletic Training*.

[13] Faelli E., Ferrando V., Bisio A. (2019). Effects of two high-intensity interval training concepts in recreational runners. *International Journal of Sports Medicine*.

[14] Mclaren S. J., Macpherson T. W., Coutts A. J., Hurst C., Spears I. R., Weston M. (2017). The relationships between internal and external measures of training load and intensity in team sports: a meta-analysis. *Sports Medicine*.

[15] Zemkova E., Oddsson L. (2016). Effects of stable and unstable resistance training in an altered-G environment on muscle power. *International Journal of Sports Medicine*.

[16] Palackic A., Suman O. E., Porter C., Murton A. J., Crandall C. G., Rivas E. (2021). Rehabilitative exercise training for burn injury. *Sports Medicine*.

[17] Azeem K. (2016). P-78 Influence of different intensities of resistance training on strength ,anaerobic power and explosive power among males. *British Journal of Sports Medicine*.

[18] Moran J., Sandercock G., Ramirez-Campillo R., Clark C. C. T., Fernandes J. F. T., Drury B. (2018). A meta-analysis of resistance training in female youth: its effect on muscular strength, and shortcomings in the literature. *Sports Medicine*.

